RETRACTED

# Tourism Demand Prediction Model Using Particle Swarm Algorithm and Neural Network in Big Data Environment

**DOI:** 10.1155/2022/3048928

**Published:** 2022-09-08

**Authors:** Sai Xu, Shuxia Wang

**Affiliations:** School of Hospitality Administration, Zhejiang Yuexiu University, Shaoxing 312000, China

## Abstract

Since demand forecasting is the first step in managing and operating a tourism business, its accuracy is very important to tourism businesses. In order to address NN's drawbacks, such as local optimization, slow convergence, and large sample sizes, this paper organically combines the PSO and NN models and builds a PSO-NN-based tourism demand forecasting model. The tourism demand forecasting indexes, the choice of NN forecasting models, the modelling process, and the implementation methods are first analysed and studied along with the fundamental theories and forecasting techniques of PSO and NN. In order to increase the precision of the prediction model, the PSO algorithm is also used to optimise the weights and thresholds of the NN. The final section of the paper compares the performance of the model developed in this paper with the most widely used model for forecasting tourism demand. According to the experimental findings, this model's prediction accuracy can reach 95.81 percent, or about 10.09 percent higher than the prediction accuracy of the conventional NN model. There are some practical implications to this research. Applying the optimization model to the forecast of tourism demand is doable and practical.

## 1. Introduction

With the development of computer network, the development of tourism is also changing rapidly: there are more and more tourism products and more varieties; travel costs are lower and travel is more convenient; even the way of traveling is quietly changing [1]. The position and role of tourism in relieving people's living pressure, improving people's living standard, stimulating domestic demand, and promoting residents' consumption are becoming increasingly prominent. The development of tourism mainly depends on the support of catering, retail, accommodation, transportation, and entertainment industries, so it is necessary to develop global tourism and attach importance to the development of tourism. At present, many regions regard tourism as the pillar or main industry of local economic development, hoping to promote the all-round development of regional economy by the development of tourism. However, with the rapid development of tourism, various problems have become increasingly prominent [2]. At present, the concept of sustainable development has gradually become the focus of tourism enterprises in various regions. Tourism practitioners must get more accurate customer needs in order to develop products that meet customer satisfaction. According to this, we should make accurate production scheduling plans, scientifically arrange transportation, accommodation, and play projects, and make the best use of available resources to get the maximum profit [3]. In this situation, it is the key for tourism enterprises in various' regions to make a good forecast of the number of tourists and their spending power. Accurate prediction of future tourism demand and establishment of corresponding mathematical model play an important role in making tourism decision-making plans [4].

RETRACTED

As a wide-ranging modern service sector, tourism has grown to be a significant factor in the growth of the national economy. The forecast of tourism demand is crucial for tourism planning. Making an effective development strategy for industries related to tourism requires accurately predicting tourism demand and researching the pattern of tourism demand from various sources. In order to better serve tourists, the government can develop effective reference strategies using the forecast trend and model of future tourism demand. The demand for tourism is always highly uncertain due to the unique characteristics of the tourism market, and any known or unknowable factors may have a significant impact on it. The statistics on tourism demand are also limited, and numerous uncontrollable factors are disrupting the market. Traditional methods have large errors, poor fault tolerance, and a lot of human factors, making it challenging to get accurate prediction results. The establishment of a reliable and workable model for forecasting tourism demand is a prerequisite for realising the sustainable and healthy development of the industry. An information processing system called a “neural network” (NN) is based on replicating the structure and operation of a biological brain's NN. It is an artificial intelligence forecasting system [5] that is data-driven. Strong nonlinear approximation, massive parallel processing, self-organization, fault tolerance, and other benefits of NN make it a useful classification and prediction tool in real-world applications. The optimization of NN has always been the focus of NN research [6–8], but it also has some flaws. The process of optimising NN structure models with intelligent optimization algorithms has been evolving and being explored in recent years with the development of these algorithms. The PSO (particle swarm optimization) algorithm is frequently used in optimization calculations because it is an intelligent optimization algorithm. In this study, a PSO optimization NN-based forecasting model for tourism demand is developed. The following are the innovations of this paper:

1. In order to address NN's drawbacks, such as the local optimum, slow convergence, and large sample size, this paper organically combines the PSO and NN models and builds a PSO-NN-based tourism demand forecasting model. The weights and thresholds of the NN are simultaneously optimised using the PSO algorithm, which has a higher prediction accuracy than other methods currently in use.
2. This study will adopt the research methods of combining theory with demonstration, quantitative, and qualitative analysis, establish the model based on the theory, and at the same time explain and support the theory with the results of the model. The method is scientific.

RETRACTED

According to the needs of research, this paper is divided into five sections. The contents of each chapter are as follows: Section 1 is the introduction. This part introduces the related research background, significance, and innovation of the research.  Section 2 is a summary of the related literature and introduces the innovation and research methods based on these related literature.  Section 3 mainly discusses the construction of related theories and models. In Section 4, the model in this paper is analysed by experiments and compared with other models.  Section 5 summarizes the content of this paper and points out the direction of further research.

## 2. Related Work

Olivé et al. used PSO with inertia weight to train NN and applied traditional genetic algorithm and PSO-NN to load forecasting [9]. The conclusion shows that PSO algorithm is the fastest and easiest way to train NN. Wen et al. established the seasonal ARIMA prediction method to predict the tourist flow of specific destinations [10]. The results show that the method has high prediction accuracy. Oc and St break the traditional constraint input from the perspective of the nonlinear relationship between the time input and the initial value of the GM model, uses PSO to solve the nonlinear problem of the time-corresponding function and finds its optimal value, and applies the model to the data forecast [11]. Vetitnev et al. will have a PSO-optimised NN with inertial weights [12]. The experimental results show that the algorithm has good convergence. Gunter and Önder select the influencing factor indicators of tourism demand from the traditional perspective and the perspective of tourism supply chain, then establish a tourism demand forecasting model according to the angle indicators with good grey correlation, and select a demand forecasting model suitable for his research according to the simulation results [13]. Untong et al. train the NN with PSO algorithm and compares it with genetic algorithm [14]. The results show that the learning algorithm of PSO-NN is simple, easy to implement, and can quickly converge to the optimal solution. Serra et al. used the combined model of NN and ARIMA model to comprehensively analyse and predict the change trend of tourist arrivals [15]. Coshall et al. conducted an empirical analysis of tourist traffic using six different forecasting techniques [16]. The results show that the ARIMA forecasting method has the strongest predictive power. Wang et al. trained the NN with the PSO algorithm and two improved PSO algorithms [17]. The conclusion shows that the PSO algorithm enhances the generalization ability of the NN. In his research on tourism forecasting methods, Gatt and Falzon pointed out that whether a single forecasting technique or a fusion forecasting technique is used, the interaction of socioeconomic conditions between the source and destination must be fully considered [18].

RETRACTED

When the corresponding assumptions are met, traditional prediction technology is more reliable, but the input set of the model is still restricted to the lag observation data of the predicted variables themselves or the factors that have an impact on the predicted variables. This paper develops a forecasting model for tourism demand based on an in-depth analysis of the PSO and NN. In this study, the initial weights and thresholds of the network are discovered by enhancing PSO, which is used to optimise the NN model. The PSO-optimised weights and thresholds are then trained using the NN algorithm, and the final model is created using these weights and thresholds. According to the research, this method has a higher prediction accuracy than the ones currently in use.

## 3. Methodology

### 3.1. Related Theoretical and Technical Basis

Exploring the tourism market, developing tourism resources, and planning and building tourist areas are all of utmost importance [19]. To do this, one must carefully examine the variables that affect tourism demand and look for the market's relevant laws of demand. Traditional linear forecasting methods frequently fail to accurately predict the complex nonlinear system that is the tourism demand. In contrast to other industries, tourism is more vulnerable to different macro- and micro-environments. To distinguish the related factors that influence tourism demand and to obtain first-hand statistical data is currently very challenging. The structure and operation of the biological brain's neural network (NN) are mimicked by the information processing system known as the NN. It is a forecasting technology for artificial intelligence that is data-driven. The NN is an example of a black-box learning technique that can automatically summarize the current data rules and determine the underlying laws of the data without relying on any empirical formula. The traits of this system include good fault tolerance, distributed information storage, and large-scale parallel processing [20]. The NN also exhibits the traits of self-organization, self-learning, and self-adaptability. The forecasting technology has been widely used in a variety of forecasting fields for social and economic activities and has achieved outstanding results in many practical application fields. This is due to its excellent self-learning performance, which still allows it to process nonlinear and incomplete data with good accuracy. The NN differs from conventional computers and artificial intelligence in that it shares many traits with human intelligence. A single neuron has a very limited function, but many neurons working together in parallel to process information together have a very strong function.  Figure 1 displays the structure of the NN.

RETRACTED

The grey system theory, which belongs to a small sample prediction and does not have to follow the typical distribution, is a method to study the issues of little data, poor information, and uncertainty. The grey NN effectively combines the benefits of good fault tolerance and strong robustness of the NN, in addition to the advantages of “less data modelling” and long-term trend modelling of the grey prediction model. As a result, the grey NN technology has many advantages over other approaches in the forecasting of tourism demand. In order to predict tourism demand accurately, one must not only minimise fluctuations brought on by unpredictable factors interacting at random but also solve the issue of incomplete data [21]. By accumulating a small number of sample data points, the grey prediction method can reduce the impact of random interference. The accumulated sequence displays a monotonic increasing trend, which can better predict the overall trend. A structured forecasting technique based on the grey system theory is the grey forecasting model. The grey series prediction model is one of many grey prediction techniques, and it predicts time series variables. The increasing rate is a feature and function of the time series-based grey series prediction model. The development of the NN has significantly increased prediction accuracy, but it also has flaws of its own. For instance, when the network is first evolving, the weights and thresholds are highly randomised, the network is prone to local optimum, and the associated parameters are fixed.

The robustness, universality, and effectiveness of the intelligent optimization algorithm make it a popular choice for the super-parameter optimization of models. Modern heuristic algorithms, which are intelligent optimization algorithms, typically have good global optimization capabilities and are appropriate for parallel processing. Theoretically, they can locate the ideal solution in a predetermined amount of time and typically have strict theoretical foundations. Based on this, this paper suggests a prediction model based on the PSO to optimise the NN, building on the current idea of integrating an intelligent optimization method with the NN in order to further increase the prediction accuracy. In biological groups, there has always been interaction between individuals and between individuals and groups. This type of behaviour demonstrates an information-sharing mechanism in biological groups, and the PSO algorithm simulates this type of social behaviour. Using this mechanism, individuals can benefit from one another's experience and advance the growth of the entire group. A popular global search algorithm used in optimization calculations is the PSO. The fundamental concept behind the PSO is to express the ideal solution to the optimization problem using the data present in each particle. A fixed optimization function determines a particle's fitness, and the particle's movement velocity vector determines the direction and length of its flight. Then, based on the current optimal particle, all particles perform a search in the potential solution space. The combination of the PSO and NN has received a lot of attention as the artificial intelligence technology has advanced. The benefit of using an intelligent optimization algorithm to optimise the NN structure is that the process does not require human involvement and can automatically design NN weights and thresholds. The acceleration constant, inertia weight, and flight speed are the three primary performance indicators for PSOs. Consequently, one optimization technique to enhance algorithm performance is parameter optimization.

RETRACTED

### 3.2. Construction of the Tourism Demand Forecasting Model

The drawbacks of the NN include slow convergence and settling into local optimum. The PSO benefits from straightforward calculations, quick convergence, high robustness, and potent global search capabilities. Currently, the NN optimised by the PSO has been used in fields such as fault detection and data compression. In this study, the PSO is used to optimise the NN model's parameters. In order to effectively address the issues with the network's weak robustness, initial value, learning rate, and momentum, we apply it to the predicted demand for tourism. We need to be able to faithfully represent the dynamic dependencies present in time series in order to build a mathematical model. To forecast the change and trend of the sequence's future direction, we identify its internal dependencies. Forecasting the demand for tourism involves taking into account a variety of factors because the tourism sector connects so many different types of industries. The nonlinear properties of the NN are used to approximate a time series in the data-driven NN model of tourism demand. The value of the past moment is used to express the value of the future moment through the obvious logical relationship of the NN. Particles should be encouraged to move throughout the entire search space in the early stages of population-based optimization rather than congregating near the local extremum. On the other hand, improving the rate of convergence of the optimal solution and successfully locating the optimal explanation are crucial in the late stages of optimization. The particle swarm optimization should, in general, be better at searching early in flight and have greater self-learning and smaller social-learning abilities. It is anticipated that as iteration times increase, especially in the later stages of flight, the ability to develop, learn socially, and self-learn will all improve. Therefore, it is necessary to evolve the learning factors and inertia weights dynamically in order to satisfy the requirements of the particle ability. The PSO-NN process is shown in Figure 2.

The diversity of the particle population will gradually deteriorate during the iterative optimization process, and there will be less room for the particles to find solutions. Simply put, the concept of mutation fixes this flaw, makes it possible for particles to locate the ideal position in a larger area, and enhances the algorithm's capacity for optimization. In this study, a new PSO parameter adaptive strategy called the dynamic acceleration constant is used. The new algorithm's goals are to promote particle movement across the entire search space in the early stages of optimization and to accelerate convergence to the best solution in the late stages of optimization. The fundamental tenet of the grey relational analysis method is to compare the sequence curve shapes of the influencing factors and the behaviour characteristics of the system under study in order to assess the degree of correlation between them. The correlation degree increases with closer curve proximity and decreases with decreasing proximity, respectively. The primary and secondary order among many influencing factors can be distinguished through the grey correlation degree, the grey correlation order, and the dominant analysis. The grey relational analysis can therefore be used to evaluate the primary influencing factors and characteristics in the study of tourism demand. The learning factor is typically set at a constant of 2 in general applications. However, dynamic evolution needs to be set up in order to serve its intended purpose. Asynchronous time-varying and synchronous time-varying are the two methods for setting learning factors. A change mode called time-varying synchronisation causes the synchronisation of two learning factors to linearly degrade. Asynchronous time-varying refers to the process of having two learning factors change over time in different ways. Its goal is to force particles to converge to the best solution at a later stage and to strengthen the global search at the beginning of optimization. The problem of how to choose the network scale when the sample size is known can be attributed to the fact that the number of samples in research on tourism demand forecasting is fixed.

RETRACTED

In order to make the data series comparable, the data should be tempered without measure. The processing methods mainly include initial value generation, average value generation, and (0, 1) interval value generation. In this paper, the initial value generation method is adopted, and the method is as follows:

(1) $$\begin{array}{c} x_{i}^{\prime }\left(k\right)=\frac{x_{i}\left(k\right)}{x_{i}\left(1\right)},i=0,1,2,3,\ldots ,m,k=1,2,3,\ldots ,n. \end{array}$$

Let *X*_0_ be the reference sequence of data behaviour, that is, the statistical data of tourism demand over the years:

(2) $$\begin{array}{c} X_{0}=\left\{x_{0}\left(1\right),x_{0}\left(2\right),x_{0}\left(3\right),\ldots ,x_{0}\left(n\right)\right\}. \end{array}$$

The grey absolute correlation degree is the reference quantity of geometric similarity between reference sequence and behaviour sequence:

(3) $$\begin{array}{c} \varepsilon_{oi}=\frac{1+\left|s_{o}\right|+\left|s_{i}\right|}{1+\left|s_{o}\right|+\left|s_{i}\right|+\left|s_{i}-s_{o}\right|}. \end{array}$$

Among them,

(4) $$\begin{array}{c} \left|s_{i}\right|=\left|\sum_{k=2}^{n-1}x_{i}^{0}\left(k\right)+\frac{1}{2}x_{i}^{0}\left(n\right)\right|,\\ \left|s_{i}-s_{0}\right|=\left|\sum_{k=2}^{n-1}\left(x_{i}^{0}\left(k\right)-x_{0}^{0}\left(k\right)\right.+\frac{1}{2}\left(x_{i}^{0}\left(n\right)-x_{0}^{0}\left(n\right)\right)\right|. \end{array}$$

*x*_0_^0^ and *x*_*i*_^0^ are the initial zeroing images of *X*_0_ and *X*_*i*_. The updated formula of particle velocity is

(5) $$\begin{array}{c} v_{\text{id}}^{k+1}=wv_{\text{id}}^{k}+c_{1}r_{1}\left[p_{\text{id}}-z_{\text{id}}^{k}\right]+c_{2}r_{2}\left[p_{g\;d}-z_{\text{id}}^{k}\right]. \end{array}$$

Inertia weight *w* plays a role in balancing global and local optimal capabilities. Its form is usually

(6) $$\begin{array}{c} w=w_{\max}-k\cdot \frac{w_{\max}-w_{\min}}{k_{\max}}, \end{array}$$

where *w*_max_ and *w*_min_ are the maximum and minimum values of weights, *k* is the number of current iterations, and *k*_max_ is the maximum number of allowed iterations. *w* can adjust the global and local search ability.

RETRACTED

When each particle searches, it takes into account the individual extremum searched by itself and the individual extremum of other particles in the group and changes its position on this basis. The transformation formula is as follows:

(7) $$\begin{array}{c} \upsilon_{i\;D}^{k+1}=\omega \upsilon_{k\;D}^{k}+c_{1}\xi \left(p_{i\;D}^{k}-x_{i\;D}^{k}\right)+c_{2}\eta \left(p_{g\;D}^{k}-x_{i\;D}^{k}\right),\\ x_{i\;D}^{k+1}=x_{i\;D}^{k}+\upsilon_{i\;D}^{k+1},\\ i=\left\{1,2,3,\ldots ,n\right\}, \end{array}$$

where *ω* is the inertia weight, and its size determines how much the particle's current speed is inherited. Appropriate selection can make particles have a balanced search ability and development ability. *k* is the current iteration number; *c*_1_ and *c*_2_ are learning factors, which are generally nonnegative constants. The learning factor enables the particle to have the ability to self-summarize and learn from the outstanding individuals in the group, and it usually takes the value *c*_1_=*c*_2_=2; *ξ* and *η* are pseudorandom numbers distributed between 0 and 1.

The speed of the particles has an impact on the optimization ability of the algorithm. Too fast speed may cause the particles to cross the optimal position, and too slow speed will make it unable to completely optimise in the population space. Therefore, it is necessary to limit the speed of the particle flight. In this paper, the maximum value *v*_max_ and the minimum value *v*_min_ of the speed are set, and the value range of the corresponding setting position *z*_*i*_ is *z*_min_ ~ *z*_max_. After training, the NN established a mapping, which is an approximation of the mapping from the previous feature space to the decision space. When making grey correlation analysis on a practical problem, we usually only consider its standardization and proximity, because some problems only need to compare the influence of multiple related factor sequences on the main sequence of the system, so we do not have to consider the other two attributes.

From the perspective of integration model construction, the GM model can make up for the uncertainty in tourism demand forecasting and give full play to the advantages of trend modelling; the NN model takes advantage of its nonlinear prediction. Finally, according to the dynamic PSO, the defects of the NN are made up. Through the construction of the fusion model, the advantages of the fusion model can be brought into full play, which can greatly improve the effect of tourism demand forecast.

RETRACTED

## 4. Result Analysis and Discussion

In the experiment, the prediction model is trained from the training set of patent authorization data, and then the prediction model is checked by using the checking data set. The newly constructed model is set with four input variables and one output variable, and the hidden layer of the network uses multilayer deep learning mode. In the PSO, the learning factors are set to be 0.5 and 2.5, and the maximum value of inertia weight is 0.9 and the minimum value is 0.1. The grey NN prediction error corresponding to the individual is taken as the individual fitness value. The population size is set to 50, the particle dimension is 4, and the number of iterative evolutions is 150. The experimental environment is based on the MATLAB development software, NN toolbox, written IPSO model, GM model, and other MATLAB programs, computer configuration: Inteli5 processor 2.90 GHz, memory 16.00 GB, 32-bit operating system, and Win7 Ultimate Edition. Under the PSO, the variation of the optimal individual fitness value with the number of evolutions is shown in Figure 3.

According to the basic viewpoint of tourism science, the main factors that affect tourism demand include national income, leisure time, physical condition, and socioeconomic condition of tourist destinations and tourist motivation. This section uses different models to forecast the tourism demand of a certain place, and the specific results are shown in Table 1.

According to the prediction results of different models in the table, it can be seen that the newly built prediction model has higher prediction accuracy than other prediction models. At the same time, it can also be found that different models show different characteristics in the process of data prediction, and the traditional NN prediction needs more training sets, so the effect is better. Therefore, we can try to find the best traditional NN to predict by cross-checking. The advantage of GM (1, 1) model is that the amount of data is small and the prediction effect of regular data is better.

In order to avoid the influence of abnormal points and the magnitude of different variables on the prediction results, the experimental data sets are standardized. The fitting curves of the established prediction model on the training set and the test set are shown in Figure 4.

The established model has a good fitting effect across the entire sample interval and strong generalization ability, as can be inferred intuitively from the trend in Figure 4, but the actual prediction effect still needs to be predicted and tested. In this study, a straightforward mutation operator is added to reinitialize the particles with a predetermined probability. The optimization is then performed by cyclic iteration until the maximum number of iterations is reached, at which point the ideal individual fitness value is recorded. The training mistakes for various models are displayed in Figure 5.

RETRACTED

The grey NN structure is determined by the dimension of input and output data. In the example study, the input data is 5-dimensional and the output is 1-dimensional. According to the principle of the grey NN, the forecast of the number of tourists based on the grey NN of the PSO is realized in MATLAB.  Figure 6 shows the linear fitting between the predicted value and the actual value.

The improved PSO-NN prediction model has more advantages than other models, as can be seen more clearly from the regression fitting between the predicted data in Figure 6 and the real data. This demonstrates that both the prediction effect and prediction accuracy are improving. From a statistical perspective, it is necessary to compare and analyze the performance measurement index and significance test to determine whether the prediction performance of the established model differs significantly from that of the benchmark model. A model must pass a number of tests to determine whether it is a valid model and whether the outcome of the next step can be predicted. The accuracy of the prediction results is one of the factors to be evaluated, and many academics assess and gauge it by the error between the predicted value and the actual value. This paper uses MSE (mean squared error), MAE (mean absolute error), and MAPE (mean absolute percentage error) as the evaluation criteria of the prediction model in order to assess the prediction impact of the newly constructed model on tourism demand. The experimental outcomes for performance indexes prediction are displayed in Table 2.

From the error data in the table, it can be seen that the error between the predicted value and the actual value obtained by this method is small, and the overall results are similar. This result shows that it is feasible to use this method to forecast tourism demand. The prediction accuracy of different models is shown in Figure 7.

It is clear that this model's prediction accuracy is higher than that of other prediction models, demonstrating the superiority of its models' prediction accuracy. The prediction accuracy of this model can reach 95.81 percent through the experimental validation in this chapter, which is roughly 10.09 percent higher than that of the conventional NN model. The prediction model developed in this paper can overcome issues with poor learning stability, low reliability, and easy NN local minima entrapment and can offer better approximation effect and faster convergence speed.

RETRACTED

## 5. Conclusions

Tourism has received increasing attention in recent years as the tertiary industry's centre of gravity, and it also contributes significantly to the growth of the national economy. The crucial link between emergency management and tourism safety is the use of scientific forecasting of tourist demand. However, the tourism sector is extremely fragile and sensitive to changes in the outside environment, and these factors, along with seasonal variations, have a significant impact. As a result, the tourism demand curve frequently exhibits complex nonlinear characteristics, making traditional forecasting techniques frequently ineffective. This paper offers a PSO-optimised NN-based tourism demand forecasting model in accordance with the current state of tourism demand forecasting. The weights and thresholds of the NN are optimised in this paper using the PSO. The inherent flaws of the NN model are somewhat overcome and the model prediction error is significantly decreased by optimising the NN with an intelligent optimization algorithm. The experimental findings demonstrate that this model's prediction accuracy can reach 95.81 percent, or about 10.09 percent higher than that of the conventional NN model. The forecasting accuracy for tourism demand can be effectively increased using this new technique. The model developed in this paper can explore the intricate linear and nonlinear properties underlying the tourism demand series in greater depth, significantly enhancing the model's ability to predict future demand. This study has some application in the real world. The optimization model can be used to forecast tourism demand in a way that is both practical and realistic. The future research focus will be on fully analysing the predicted effects of six factors (clothing, food, housing, transportation, entertainment, and purchases) on tourism.

## Figures and Tables

**Figure 1:** NN structure.

**Figure 2:** PSO-NN process.

**Figure 3:** Dynamic PSO optimization process.

**Figure 4:** The fitting effect of this model on training set and test set.

**Figure 5:** Training errors of different models.

**Figure 6:** Linear fitting between predicted value and actual value.

**Figure 7:** Prediction accuracy of different models.

**Table 1:** Prediction results of different models.

Date	True value	Traditional NN model	GM model	Model of this paper
2021/1	256397	251756	257443	259520
2021/2	124289	143074	271532	125864
2021/3	213895	132586	241240	220634
2021/4	243971	239629	242785	247586
2021/5	352976	337376	296127	368747
2021/6	344905	254130	304798	337469

RETRACTED

**Table 2:** Experimental results of predicting performance indicators.

Methods	MSE	MAE	MAPE
The traditional NN model	16.87	3.27	0.084
The GM(1, 1) model	13.21	2.14	0.071
AdaBoost-ELM	12.14	2.85	0.067
Optimization model in this paper	12.08	2.13	0.063

## Data Availability

The data used to support the findings of this study are available from the corresponding author upon request.
